The article "A Case Report of Spindle Cell (Sarcomatoid) Carcinoma of the Larynx" was published in 2012. Journal: Case Rep Med.

# A Case Report of Spindle Cell (Sarcomatoid) Carcinoma of the Larynx

**DOI:** 10.1155/2012/370204

**Published:** 2012-12-20

**Authors:** Harry Boamah, Billy Ballard

**Affiliations:** ^1^Meharry Medical College, 1005 DR DB Todd Boulevard, Nashville, TN 37208, USA; ^2^Department of Pathology, Meharry Medical College, 1005 DR DB Todd Boulevard, Nashville, TN 37208, USA

## Abstract

Spindle cell carcinoma (SpCC) or sarcomatoid carcinoma is a highly malignant variant of squamous cell carcinoma which comprises 2% to 3% of all laryngeal cancers. It is considered to be a biphasic tumor that is composed of a squamous cell carcinoma (in situ or invasive) and spindle cell carcinoma with sarcomatous appearance. Most spindle cell tumors are polypoid and pedunculated; they are often detected at an early stage, removed by polypectomy during diagnosis, and tend to have a very good prognosis. We present a case of spindle cell carcinoma in a 67-year-old Caucasian male who presented with progressive hoarseness of his voice, dysphagia, odynophagia and a 20-pound weight loss. The patient underwent direct laryngoscopy with excision of the malignant mass and received radiation therapy. His symptoms gradually improved, and he regained good control of his voice.

## 1. Introduction

Spindle cell (sarcomatoid) carcinoma of the larynx is a rare tumor and comprises 2% to 3% of all laryngeal cancers [1]. Squamous cell carcinoma is the most malignant carcinoma of the larynx, and spindle cell (sarcomatoid) tumor is considered a highly malignant variant of squamous cell carcinoma. Spindle cell carcinoma is considered to be a biphasic tumor that is composed of a squamous cell carcinoma (in situ or invasive) and spindle cell carcinoma with sarcomatous appearance [2]. Since a majority of these tumors are polypoid or pedunculated and tend to cause obstructive symptoms, these tumors are often detected at an early stage, removed by polypectomy during diagnosis, and tend to have a very good prognosis. The following is a case report of one such patient who presented to our institution with spindle cell (sarcomatoid) carcinoma of the larynx.

## 2. Case Report

A 67-year-old Caucasian male presented to the internal medicine clinic with 2-month history of progressive hoarseness that has been affecting his ability to speak and dysphagia. The patient also described a 20-pound weight loss over the last several months due to his dysphagia and odynophagia. The patient history was significant for 60 packs years of smoking.

In the clinic, the patient had difficulty in speaking and hoarseness of in voice. Physical examination of the patient showed a very small palpable lymphadenopathy in the anterior cervical region more pronounced on the right compared to the left. The patient did not have any supraclavicular lymph nodes bilaterally.

The article "A Case Report of Spindle Cell (Sarcomatoid) Carcinoma of the Larynx" was published in 2012. Journal: Case Rep Med.

A CT scan of his neck with contrast revealed a 7 mm polypoid mass involving the anterior commissure of the vocal cords; however the nasopharynx, pharynx, peripharyngeal spaces and epiglottis appeared unremarkable. The parotid gland and submandibular salivary glands were normal; however the CT showed that the thyroid gland was enlarged. There was no adenopathy noted however (Figure 1).

The patient underwent a flexible laryngoscopy that showed the presence of an anterior commissure mass. The patient then underwent direct laryngoscopy with biopsy, rigid bronchoscopy, and esophagoscopy which showed a pedunculated mass located in the anterior commissure with extension of the pedunculated portion into the glottic and subglottic regions. The lesion of the pedunculated mass was biopsied for pathology. 

The pathology report showed a spindle cell (sarcomatoid) carcinoma (Figure 2) that strongly stained for EMA, CK 5/6 and AE 1/3, and a high MIB-1 but negative for myoD1, SMA, desmin, and myf4 (Figure 3).

The patient underwent a positron emission tomography scan of the full body which showed FDG avidity in the anterior larynx with SUV of 3.6 consistent with his vocal cord mass but no increased FDG avidity within the neck. There was also an increase in FDG avidity with SUV 6 in the right paratracheal region of concern for a second primary malignancy. However a CT scan of his chest did not show any mediastinal mass or lymphadenopathy.

The patient spindle cell (sarcomatoid) carcinoma was staged T1 because the tumor was pedunculated and attached only at the anterior commissure even though it prolapsed into the glottic and subglottic region of the vocal cord.

The patient was evaluated by head and neck surgery, and his tumor was found to be amenable to surgical excision and adjuvant radiation therapy. The patient underwent direct laryngoscopy with excision of the malignant mass and received radiation therapy. The patient's symptoms gradually improved, and he regained good control of his voice.

## 3. Discussion

Squamous cell carcinoma (SCC) is considered to be the most common type of malignant laryngeal tumor [1]. Spindle cell carcinoma (SpCC) or sarcomatoid carcinoma is a highly malignant variant of squamous cell carcinoma. It is a rare tumor with a reported incidence of 2% to 3% of all laryngeal cancers [2]. Spindle cell carcinoma is considered to be a biphasic tumor that is composed of a squamous cell carcinoma (in situ or invasive) and spindle cell carcinoma with sarcomatous appearance [2]. SpCC is also considered to be a monoclonal epithelial neoplasm with the sarcomatous component derived from squamous epithelium with divergent mesenchymal differentiation [2]. Although the exact cause of SpCC is not known, it is strongly associated with a history of cigarette smoking and alcohol abuse. It has also been suggested that SpCC is associated with radiation exposure although the determination of radiation risk may be complicated by the dose and duration of radiation exposure [3]. SpCC is more predominant in men compared to females (12 : 1 ratio) although it is becoming more common in females, and it is usually seen in the 6th and 7th decades of life [4]. 

The article "A Case Report of Spindle Cell (Sarcomatoid) Carcinoma of the Larynx" was published in 2012. Journal: Case Rep Med.

Spindle cell carcinoma most commonly affects the glottis in the majority of cases (70%), and the majority of patients present with symptoms of hoarseness, dyspnea, cough, and dysphagia often of less than 1-year duration [1]. The majority of these tumors are characterized as being polypoid or pedunculated (98.9%) tumors that are often less than 2 cm in size [4]. The diagnosis of spindle cell carcinoma requires histological demonstration of both the squamous cell component and the spindle shape cells with sarcomatous appearances [2]. Histological examination can often show the presence of squamous cell carcinoma at the surface or deeper within the tumor although this is rare especially with tumors where the surface is ulcerated or denuded. What is often seen is a blending of squamous cells and spindle cells which can be differentiated by their different arrangement which includes storiform, solid, and fascicular appearance [4]. In about half of cases there is also a desmoplastic stromal fibrosis, and because the epithelial cells are capable of transforming into sarcomatoid spindle cells, it is not uncommon to see the presence of bone and cartilage and or osteosarcoma and chondrosarcoma on histology. 

In addition to histological studies, immunohistochemical studies of epithelial and mesenchymal markers are used to diagnose the tumor. Epithelial markers include keratin (AE1/AE3, CK1, 8, 9), epithelial membrane antigens, KI, and K18. Mesenchymal markers include vimentin, desmin, S-100, Osteopontin, and BMP (2, 4) [5]. For spindle cell carcinomas with poorly differentiated epithelial tumor components Lewis et al. have shown that p53, a transcription factor that is important for epithelial proliferation and differentiation, isparticularly useful for diagnosing SpCC of the head and neck region [6]. 

Spindle cell carcinomas are staged according to the TNM classification scheme of the American Joint Committee on Cancer staging. Tumors are staged according to their size and the presence or absence of metastasis to local lymph nodes or other parts of the body [3]. The treatment of spindle cell carcinoma is most influenced by the tumor location and the stage of the tumor including tumor metastasis. Other factors that are important include laryngeal preservation, good voice control posttreatment, and a lower risk of treatment complications [4]. Tumor size, locations (supraglottic, glottis, or subglottic), vocal cord mobility, and tumor stage can all impact the treatment and outcomes of patients. The majority of spindle cell tumors are detected early in stages T1 and T2 due to their obstruction of the larynx causing symptoms and are correlated with a better prognosis [4]. Since most spindle cell tumors are polypoid and pedunculated, polypectomy and wide local excision during diagnosis can completely eliminate the entire tumor mass because of their noninvasion of the underlying stroma at that early stage [3]. Tumors that are stage T2 or less can be managed conservatively with limited field irradiation and conservative treatment to preserve the patient's voice. Tumors that are stage 3-4 can be treated with local resection, partial laryngectomy, total laryngectomy with or without lymph node dissection followed by combination of radiation therapy and chemotherapy [4]. Spindle cell carcinoma of the larynx has a very good 5-year prognosis of 65%–95% [1]. Poor prognostic factors include tumors diagnosed at higher stages, large tumors (>3 cm) with a predominance of epithelial component, nonglottic tumors, fixed vocal cords, history of radiotherapy and metastasis to regional lymph nodes, and distant metastasis [4].

The article "A Case Report of Spindle Cell (Sarcomatoid) Carcinoma of the Larynx" was published in 2012. Journal: Case Rep Med.

## 4. Conclusion

Spindle cell carcinoma (SpCC) or sarcomatoid carcinoma of the larynx is a highly malignant variant of squamous cell carcinoma that is very uncommon. Because most spindle cell tumors are polypoid and pedunculated and tend to cause obstructive symptoms such as hoarseness, dyspnea, and dysphagia, most tumors without metastasis are detected early and tend to have a very good 5-year prognosis. 

This patient's spindle cell (sarcomatoid) carcinoma was staged T1NO without any evidence of metastasis. Due to the early detection of the tumor, the patient underwent surgical excision and adjuvant radiation therapy. His symptoms subsequently improved, and he regained good control of his voice.

## Figures and Tables

**Figure 1:** CT of the neck with contrast: There is 7 mm polypoid mass involving the anterior commissure of the vocal cords. The nasopharynx, and pharynx, peripharyngeal spaces appear unremarkable, as well as the parotid and submandibular salivary glands. There is no significant neck adenopathy noted.

**Figure 2:** Histological findings: loose myxomatous fibrous connective tissue containing both spindle-shaped cells as well as ovoid cells with hyperchromatic, pleomorphic nuclei with eosinophilic cytoplasm. In some areas, cells assumed a whirling interlacing pattern and at one margin dysplastic-stratified squamous epithelium characterized by cells with pleomorphic hyperchromatic nuclei.

The article "A Case Report of Spindle Cell (Sarcomatoid) Carcinoma of the Larynx" was published in 2012. Journal: Case Rep Med.

**Figure 3:** Immunohistochemistry: cytokeratin AE1/AE3, strongly positive diffuse nuclear staining of neoplastic cells, Ck 5/6, strongly positive nuclear cytoplasmic staining of neoplastic cells, vimentin, strongly positive. Epithelial membrane antigens (EMA) was positive.
